The article "Influence Mechanism of Educational Leadership on Environmental Accounting Based on Big Data Algorithm" was retracted in 2023. Reasons: unreliable results or conclusions; concerns about the data; concerns about the peer review; concerns about the citations.

# Influence Mechanism of Educational Leadership on Environmental Accounting Based on Big Data Algorithm

**DOI:** 10.1155/2022/5690230

**Published:** 2022-10-06

**Authors:** Minyan Jin, Li Yao

**Affiliations:** ^1^College of Accounting, Zhanjiang Science and Technology College, Zhanjiang, 524009 Guangdong, China; ^2^School of Human Science, Assumption University, Bangkok 10240, Thailand

## Abstract

Over the last 20 years, big data techniques in teaching have been overgrown. Making educational decisions now includes information knowledge as a crucial component. This started a trend for using big data algorithms strategically. Technological advances have been used to analyze the enormous amount of information and develop strategic judgments. The current study aims to address issues with the conventional instructional, administrative management solution focused on manual rule formulation in big data storage and interpretation and has poor efficiency in analyzing big data and lacking value in developing education leadership qualities. The study suggests an educational leadership model based on big data algorithm (ELM-BDA) to explore the student leadership performance that relies on cooperative filtration and fuzzy C-means (FCM) and big data. The different influencing mechanisms and factors directly linked to educational leadership were also analyzed using a big data algorithm. To build an intelligent institutional administrative system, the research also exposes it to organizational studies. By evaluating the big data research already in existence, this study emphasizes the expanding significance of big data. Additionally, this study explores the effects of big data analytics on educational leadership qualities by utilizing an FCM. A scoring system is designed to predict the student's leadership level, and using the big data algorithms, the students are motivated and trained to improve their skills. The education and learning method can be enhanced at educational institutions through better decision-making to use this big data for leadership development. Big data facilitates efficient educational decision-making by merging various data and telecommunications technologies. Using big data in schooling will increase—leadership quality among students. To effectively use big data for decision-making, academic leaders must create new types of learning and monitoring systems.

## 1. Introduction to Educational Leadership

Many initiatives have attempted to evaluate and analyze the performance of education leadership management in elementary, secondary, and university education tiers worldwide. The qualities, behaviors, and styles of leaders were the subject of several studies, but it is still essential to examine how each factor contributes to strong leadership. The main goal of this study is to explore the relationships between these fundamental elements and the efficacy of administration concerning them. The development of an adequate evaluation tool for evaluating the effectiveness of education management using measurements and criteria related to the activities and behaviors of leaders is another target of this research.

The article "Influence Mechanism of Educational Leadership on Environmental Accounting Based on Big Data Algorithm" was retracted in 2023. Reasons: unreliable results or conclusions; concerns about the data; concerns about the peer review; concerns about the citations.

From ancient times to the present, humanity has been preoccupied with the question of management and its effects. Researchers, academics, scientists, industry and affiliation executive officers, private and general populace sector managers, politicians and authorities, structured communities and informal institutions, military installations, and educational establishments have all given it some thought. The notion of leadership has occasionally been interpreted and analyzed based on the traits of the leader's character on the foundation of the outcomes and the commanding style or with “hybrid” frameworks that mix the management and academic models. Additionally, schools routinely examine various initiative variables that significantly impact academic success to assess the reform process [1].

By connecting the efficacy of management with the traits of the managers, the leadership styles, their behaviors, and the linkages between them, this study is aimed at fostering reflection and drawing conclusions about education leadership management.

Over the past few years, there has been an increasing trend toward creating learning solutions for processing big data [2]. Learners worldwide are now using smartphones' web content due to the advent and quick growth of the internet. Their online activities produce a vast amount of information that can be gathered using various technologies. This enormous volume of data is used to provide helpful information when making decisions about schooling.

Researchers define big data in several ways [3]. In teaching, “big data” refers to the practical analysis of huge amounts of information to provide helpful knowledge [4]. This idea can fundamentally alter how it handles the educational process by changing how students and teachers connect and effectively meeting every learner's unique needs [5]. Typically, there are a variety of questions about leadership and government, such as whether something is efficient, what qualities define it as efficient, if the traits of the ruler or the management style study its effect, or more purely when a manager is able or willing to do something. Environmental accounting is a field that identifies the environmental factors that affect the nation's economy. Educational leadership is defined as the process of guiding the talents and energies of teachers. Environmental accounting or ecological factors affect the educational context and may be applied in schools, colleges, or universities to improve student leadership skills. The study shows a strong relationship between leadership and learner performance considering environmental accounting factors. To fully incorporate environmental accounting into educational leadership, big data algorithms are needed to provide enough data for the process. The big data algorithm helps provide enormous data and fetch the required factor to enhance the education leadership skills from the available data.

The article "Influence Mechanism of Educational Leadership on Environmental Accounting Based on Big Data Algorithm" was retracted in 2023. Reasons: unreliable results or conclusions; concerns about the data; concerns about the peer review; concerns about the citations.

The primary contributions of the study are listed below:

- A leadership score prediction model for the student is designed in this research using FCM. This model is used to analyze the leadership quality present in the students, and prediction results can be increased using a big data algorithm
- The different influencing factors which affect and improve the education leadership quality are analyzed and discussed
- The implications of the big data algorithm in education leadership are discussed, and future suggestions and recommendations are enumerated in this research

The reminder of the article is organized as follows: Section 2 enumerates the background of educational leadership and its impact. The proposed educational leadership model based on big data algorithm (ELM-BDA) is designed and mathematically derived in Section 3.  Section 4 analyses and shares the proposed system's outcomes and exhibits the system's higher yields.  Section 5 illustrates the conclusion and findings of the study.

## 2. Background to the Education Leadership and Its Impact

An exhaustive relative literature analysis in education management has been conducted in this study to examine the most crucial elements of instructional leadership from top to bottom. The focus of this study is more explicit on which of these factors is thought to add more to strong leadership in educational settings—leader personal qualities, applied specific behaviors, or good leadership styles. The sole objective of this study is to establish the relevant research issues and to propose a structure for more essential elements of teacher management so that the investigations are more successful.

The relative importance of every one of the main crucial management styles, regardless of academic efficiency and the relationship between them and effectiveness, was examined in a follow-up survey using a relevant survey. Concerning teachers' perspectives as attendees and shareholders in a sample solution, the survey attempts to determine the significance of leaders' behaviors and analyze which of the above individual elements are deemed more essential and have a more significant impact on academic leader behavior. Management in education is a growingly fascinating field of study. This is due to the thorough exploration of the educational function's outcomes on the one side and the pursuit of leaders' effects on products on the other [6].

The article "Influence Mechanism of Educational Leadership on Environmental Accounting Based on Big Data Algorithm" was retracted in 2023. Reasons: unreliable results or conclusions; concerns about the data; concerns about the peer review; concerns about the citations.

Another factor that keeps people interested in the education sector is that it has become increasingly demanding as new problems for leaders emerge. Globally, the education system has come to recognize the role and importance of education institutions. It is said to play a crucial part in enhancing academic development and performance by influencing teachers' motivations and skills and the culture and community of the classroom. The usefulness and worth of tutoring can only advance with competent school management [7]. Among the most critical variables in the progression of the standard and uniqueness of a school is believed to be the school founder [8]. Education leadership can be categorized into transformational leadership, transform leadership, and decision-making leadership.

Many studies in the past have shown that the management style and skills of the principal have an impact on a range of teacher characteristics, including job contentment and efficiency, as well as levels of engagement and academic accentuation [9]. It can influence the motivation and performance of educators by creating the right mood and working environment, which significantly affects the quality of the school's outcomes [10]. Additionally, research has shown that a principal's management can have a considerable, albeit indirect, impact on students' academic performance [11–13]. The most important factor contributing to the growing importance of educational change is the rising expectations of people and organizations, both within and without the education sector and from institutions suggested by Farley-Ripple et al. [14]. Additionally, as should be clear from the reading of the pertinent literature, the many groups of people who are “included” in or benefit from any sort of academic management, such as educators, pupils, or families, depend significantly on the decisions made by the educational leaders.

Big data has made it possible for educational leadership to take prompt, efficient actions to enhance corporate culture and the educational experience for students [15]. Big data can fundamentally alter how education and study are conducted in the future. The use of data to drive teaching was among the five most comprehensive policies linked to significant educational achievements, according to a study done on 35 school choices in New York City in the United States suggested by Ray and Saeed [16].

The article "Influence Mechanism of Educational Leadership on Environmental Accounting Based on Big Data Algorithm" was retracted in 2023. Reasons: unreliable results or conclusions; concerns about the data; concerns about the peer review; concerns about the citations.

Cloud computing is a component of big data technologies. These collaboration solutions can enhance educational offerings by providing underprivileged students with the inexpensive expansion of online content [17]. Furthermore, as the author noted, big data can complement the conventional instructional system by aiding teachers in analyzing what kids know and what approaches are most successful for every pupil. As a result, it also gives teachers data on how to enhance learning by altering their classroom practices and methodologies. Moreover, learners and staff can receive fast feedback regarding their academic achievement using technologies like information analysis [18]. According to the author, such technologies aid in developing educational patterns that give educational authorities crucial information.

For instance, instructional patterns can release secrets about a student's unique needs, and by making wise choices, the risk of their failures and dropouts can be reduced. The author further claimed that these instructional patterns aid in creating unique pedagogical strategies that are effective with a specific group of pupils with special requirements.

In addition to these applications, their research indicates that big data can transform the traditional educational system into an online one suggested by Hong [19]. The use of learning systems has recently spread around the globe. More and more people are using these networks, which leads to the online creation of new data. This further information gathered through various channels assists faculty members in understanding educational requirements and emerging trends [20].

Even though there are few applications of big data in education, this trend is steadily growing. This growing tendency is caused by how well data-driven decision-making works. Academic institutions require trained personnel who can manage vast amounts of data and all these technologies as this trend is expected to intensify soon. To support the data-driven selection process, school administrators must get conversant with these new resources or create a dedicated department or position. Thus, the need for computer scientists and information analysts in the education sector is undoubtedly increasing shortly.

## 3. Proposed Educational Leadership Model Based on Big Data Algorithm

Environmental accounting is a field that identifies the environmental factors that affect the nation's economy. Educational leadership is defined as the process of guiding the talents and energies of teachers. Environmental accounting or ecological factors affect the educational context and may be applied in schools, colleges, or universities to improve student leadership skills. The study shows a strong relationship between leadership and learner performance considering environmental accounting factors.

The article "Influence Mechanism of Educational Leadership on Environmental Accounting Based on Big Data Algorithm" was retracted in 2023. Reasons: unreliable results or conclusions; concerns about the data; concerns about the peer review; concerns about the citations.

The research revealed that most students' educational leadership quality is hidden. This research aims to focus on the different education leadership affection influenced environmental parameters, and the outcomes are enhanced using a big data analytical model. The model initially analyzes and predicts the student's leadership score.

The clustering model of the proposed research is indicated in Figure 1. The study starts with clustering the students based on their leadership skills, initializing their weighting index, and then the threshold level for leadership detection is identified and initialized. Based on the cluster and cluster center of the function, the convergence of better skills for leadership is analyzed, and if not attained, the cluster initialization is repeated.

### 3.1. Influencing Factors of Education Leadership Conditions

Teaching technique design, practical assistance, and material circumstances are three factors that impact how students learn. When viewed from the standpoint of instruction, it primarily entails the creation of instructional goals and developing instructional materials, strategies, and activities. The main component influencing the learning experience is that, from the students' perspective, the teaching goals must be established in a manner that is compatible with the educational purposes of the classmates.

The education platform's publications and course materials are typically provided using graphics and film, with video serving as the primary medium. According to the survey, most students utilize their free time to learn. Thus, the teaching time must satisfy their objective needs. For instance, if the teaching time is too lengthy, the student cannot finish the learning about education leadership; however, it slows down the learner's perseverance to a specific extent, making it difficult for the learner to focus solely; conversely, if the teaching is too limited, it hurts the other edge. On the other side, learning development forces students to operate too often. The typical course video lasts 30-45 minutes.

From the standpoint of the teaching material, the selection and configuration of the teaching material can empower the learners to engage with the framework, educators, and other beginners, the video play screen, the place of the course warning, the doorway of the comment bar, the opening of the message board, the glass wherein the teacher's aide and the student talk, or if the place of these streams is sensible. The learner's ability to participate in the program depends on the video's length, clarity, and reasonableness, as well as whether or not there will be any stuttering.

The article "Influence Mechanism of Educational Leadership on Environmental Accounting Based on Big Data Algorithm" was retracted in 2023. Reasons: unreliable results or conclusions; concerns about the data; concerns about the peer review; concerns about the citations.

How well the different teaching connections, like the number of tasks, the regularity of exams, the frequency of giving answers, and how well the pedagogical practices can ultimately mobilize and enhance the students' passion are matched to the level of learners for leadership quality. Whether the job is challenging enough, whether the teaching method can accommodate the learner's smart device's learning requirements, and whether the student tries to talk via instant messenger programs to increase the viscosity among the student and the platforms, it is essential to determine if the teaching approach can successfully increase the student's internal interest in leadership. If the way of evaluating instruction can successfully assess the learner's learning methods and results, it is said to be diverse and acceptable.

### 3.2. Emotional Conditions for Leaders

Social networks between students and other students and between students and professors, and managers are all connected with learner involvement, such as attitudes and excitement for learning and systems. Whether the design of the education process, such as the different instructional links, the volume of assignments, the regularity of quizzes, the frequency of Question and Answer (Q&A), or if the learners can be fully mobilized and enhanced, can fit the requirements of the learner. If the student's enthusiasm and the level of difficulty of the assignment are compatible; if the teaching method can accommodate the student's mobile extension's educational needs; and if the student needs to talk via instant messenger program.

To increase the viscosity among the student and the platforms, it is essential to determine whether the approach to teaching can successfully motivate the student's innate drive for studying or if the learner's leadership participation is appropriately rewarded. Suppose the approach to assessing instruction is flexible, reasonable, and capable of efficiently evaluating, and the student's learning results are enhanced.

Together, instructors, administrators, and students can boost emotional involvement, and their positive interactions make students more likely to continue with their classes, platforms, and peers. The education system is promoted in many domestic and international studies, and student accomplishment levels are not scored and graded.

Nevertheless, in the education leadership environment, the primary goal of rating or marking is not to motivate students who are learning more slowly but motivating students who are learning more quickly and with more incredible excitement through the same rankings. Enhance the student's feeling of accomplishment to some level, recognize the value of learning, provide the learner with a sense of connection, and foster a healthy competitive market. The social component of the learning platform must be strengthened, and interactions between users and other players must be improved. The classroom experience falls short of the ambiance of traditional instruction in the classroom setting without a big data algorithm.

The article "Influence Mechanism of Educational Leadership on Environmental Accounting Based on Big Data Algorithm" was retracted in 2023. Reasons: unreliable results or conclusions; concerns about the data; concerns about the peer review; concerns about the citations.

The learning environment ought to make an effort to establish a higher education leadership quality among students. Together domains include panel discussions, course boards, and post bars? These environments test teachers' and supervisors' ability to manage and promptly reply to message boards and post bars, as well as the ability of students to pose teacher questions and receive timely answers, whether or not students can assist and correct one another. In addition to providing instruction, the learning platform should be able to schedule offline activities concurrently with in-person instruction to increase students' emotional engagement and leadership quality. In summary, the learner's inner driving force frequently impacts how their emotional state affects their learning experience.

While a bad impact cause students to become disinterested in their studies, lack trust, and find it challenging to solve difficulties, a positive result can encourage students to invest in their education.

### 3.3. Students' Leadership Score Expectation

The process of studying and processing the provided objects using analytical models, then, separating and categorizing them based on how similar they are to one another, is known as a clustering algorithm. With the development of fuzzy theory, individuals started applying fuzzy techniques to clustering issues, specifically the fuzzy-based study. Fuzzy grouping can handle a variety of objects where attribute differentiation is not always clear in real-world situations. To indicate the similarity among samples, the classifier is used. Fuzzy clustering represents the ambiguity of the sampling for the group, which could more accurately represent the actual world because it obtains the level of uncertainty for every classification and the sample size.

The targets are typically clustered using the fuzzy clustering technique based on empirical function using different students based on their educational leadership skills. The sample set represented is  *S* = {*s*_1_, *s*_2_, ⋯, *s*_*N*_}. The weighted function of the cluster is denoted as *β*_*yn*_. And equation (1) shows the relationship of all the cluster weighting function sum as 1. The different parameters should be weighted with varying scales of weight to find the optimum results.

(1) $$\begin{array}{c} \overset{N-1}{\underset{y=0}{\prod }}\beta_{yn}=1. \end{array}$$

*y* = 0, 1, ⋯, *N* and *n* = 0, 1, ⋯, *N*. The number of sample *S* transmitted is indicated by the variable *n*(0 ≤ *n* ≤ *N*). The parameter represents the level of sample *n*'s participation in the class *y* as *β*_*yn*_ ∈ [0, 1]. The fuzzy division matrix *M* is indicated in equation (2). The grouped students are separated, and their teaching model is varied based on the *M* value. This matrix is formed using the different environmental influencing factors *β*_*xy*_.

(2) $$\begin{array}{c} M=\left[\begin{array}{ccc} \beta_{11} & \beta_{12} & \cdots \;\beta_{1N}\\ \beta_{21} & \beta_{22} & \begin{array}{cc} \cdots & \beta_{2N} \end{array}\\ \begin{array}{c} \vdots \\ \beta_{N1} \end{array} & \begin{array}{c} \vdots \\ \beta_{N2} \end{array} & \begin{array}{cc} \begin{array}{c} \vdots \\ \cdots \end{array} & \begin{array}{c} \vdots \\ \beta_{NN} \end{array} \end{array} \end{array}\right]. \end{array}$$

The matrix is used to find the leadership quality of a student using different parameters. The degree to which the sample *S*_*n*_ belongs to class *y* is indicated by the symbol *β*_*yn*_. Currently, fuzzy C-means, which primarily determines the class of key points to categorize sample information automatically, is the most frequently used FCM. FCM obtains the membership grade of every sampling site to all category centers by optimizing the optimal solution to enhance the influencing environmental mechanisms. The function for each cluster is assigned to a sample, and the data are then categorized according to the membership functions. The object method *O*_*f*_ is represented in equation (3). The objective function is expressed as the central theme of the proposed model, which is the leadership analysis.

(3) $$\begin{array}{c} O_{f}=\overset{N-1}{\underset{x=0}{\prod }}\overset{N-1}{\underset{y=0}{\prod }}\frac{\beta_{xy}^{w}}{{\left(S_{n}^{y}-C_{c}\right)}^{2}}. \end{array}$$

The term *w* stands for a weighted index, where *w* > 1 designates the fuzzy level of the grouping outcomes. The most accurate empirical results are used, with *w* = 2. The variable *S*_*n*_ denotes sample *n* inside the source (*S*). The cluster center is characterized by *C*_*c*_, and the participation function is represented by *β*_*xy*_^*w*^.

The article "Influence Mechanism of Educational Leadership on Environmental Accounting Based on Big Data Algorithm" was retracted in 2023. Reasons: unreliable results or conclusions; concerns about the data; concerns about the peer review; concerns about the citations.

Equation (4) is used to address the constraint minimization function and make *O*_*f*_ minimal. The constraints show the limitation of the educational leadership, and the factors that influence the prediction score are constrained by 1.

(4) $$\begin{array}{c} \min\overset{N-1}{\underset{x=0}{\prod }}\overset{N-1}{\underset{y=0}{\prod }}\frac{\beta_{xy}^{w}}{{\left(S_{n}^{y}-C_{c}\right)}^{2}}\text{ where }\overset{N-1}{\underset{y=0}{\prod }}\beta_{yn}=1. \end{array}$$

The sample *n* in *S* is denoted by *S*_*n*_. The cluster center is characterized by *C*_*c*_, and the participation function is represented by *β*_*xy*_^*w*^. The total number of samples available is indicated as *N*. The logistic regression (*L*) technique resolves the issue using equation (5). *L* solves the solution for the clustering head, and the education leader is selected based on the higher *L* value.

(5) $$\begin{array}{c} L=\overset{N-1}{\underset{x=0}{\prod }}\overset{N-1}{\underset{y=0}{\prod }}\frac{\beta_{xy}^{w}}{{\left(S_{n}^{y}-C_{c}\right)}^{2}}-\overset{N-1}{\underset{x=0}{\prod }}\rho_{x}\left(\overset{N-1}{\underset{y=0}{\prod }}\beta_{yn}-1\right). \end{array}$$

*w* is a weighted index, *S*_*n*_ is a reference to samples *n* in *S*, *C*_*c*_ is the group center, *β*_*yn*_ is the participation function, *L* represents the logistic regression method, and *ρ*_*x*_ is a component multiplier. The total sample size is denoted as *N*. The partial dependencies of *L* about *C*_*c*_, *β*_*yn*_, and *ρ*_*x*_ are then brought to zero in the manner described using equation (6). The partial influencing environmental factors which are linked to educational leadership are analyzed and shown below:

(6) $$\begin{array}{c} \beta_{yn}=\frac{{\left(S_{n}-C_{c}\right)}^{2/w-1}}{\prod_{x=0}^{N-1}{\left(S_{n}-C_{c}\left(x\right)\right)}^{2/w-1}}. \end{array}$$

The terms *β*_*yn*_ and *w* denote for a membership value and weighted index, samples *n* in *S* are indicated as *S*_*n*_, and *C*_*c*_(*x*) is the group center. *N* indicates the total number of samples. The cluster center is shown in equation (7) which is used to find the optimum leadership quality among the students. The cluster center is the best student with higher education leadership quality with higher influencing environmental factors.

(7) $$\begin{array}{c} C_{c}\left(x\right)=\frac{\prod_{y=0}^{N-1}\beta_{xy}^{w}\times S_{n}}{1+\prod_{y=0}^{N-1}\beta_{xy}^{w}}. \end{array}$$

*C*_*c*_(*x*) is the group center, *w* is a weighted index, *S*_*n*_ is a reference to samples *n* in *S*, and *β*_*xy*_^*w*^ is a participation value. The total number of samples is denoted as *N*.

First, the parameters *N* and *w* are specified to represent the number of fuzzy-based categories. *i* reflects on the number of iterative processes and describes the threshold to cease iteration. The clustering center is then set up a second. To achieve the final grouping center and fuzzy partition matrices, iterative transactions are carried out during the third step, updating the membership degree and the grouping center only until the outcome converges.

The article "Influence Mechanism of Educational Leadership on Environmental Accounting Based on Big Data Algorithm" was retracted in 2023. Reasons: unreliable results or conclusions; concerns about the data; concerns about the peer review; concerns about the citations.

Using the fuzzy clustering technique, the school leadership system's data could be mined for valuable data and its underlying laws. To better understand trainees, enhance teaching, fortify management, and enhance pertinent systems, it aids in proving the effectiveness of school enrollment and jobs administration, teacher management, instructional strategic planning, learning outcomes guidelines, governance, and investment and hardware management.

A method used in systems and network filtering is the FCM algorithm. It is being used to assess students' interests, locate students in the user community who feel the same way as the particular student, combine these students' evaluations of the same material, and create a system to anticipate the student's choice for that information. It is possible to think of the forecast of students' achievement as the “recommended” of students' success, and the nearer students' test scores are to one another, the more comparable the circumstances or other factors are among them. The previous student information can be used to identify equivalent students to forecast a student's leadership success.

Students in the information retrieval of new datasets correlate to students' interests. The previous outcomes of these comparable students can be combined to forecast the success of the chosen students. The current work combines FCM and big data to suggest a model for predicting education leadership achievement.

The student education leadership performance analysis based on environmental accounting factors is indicated in Figure 2. The student data is collected from 200 boy and 100 girl students. Based on their response, they are grouped into different clusters using the cluster membership function. The education leadership is computed and predicted based on environmental factors and big data. The results are calculated using the updated weighting function using FCM and a big data algorithm.

The participation matrices of every student in every group are obtained when the historical students' academic data are first clustered using cluster analysis technology. Then, using the dispersion of every student subscribing to every group and the information retrieval approach related to students, the forecast of every cluster to anticipate students' return is measured.

The article "Influence Mechanism of Educational Leadership on Environmental Accounting Based on Big Data Algorithm" was retracted in 2023. Reasons: unreliable results or conclusions; concerns about the data; concerns about the peer review; concerns about the citations.

Finally, the proportion of the targeted candidates admitted per each cluster is weighted to produce the final predictive performance. The different leadership qualities include transformation quality, leadership quality, and decision-making skills. The following are specific forecasting methods.

The efficiency of student-*st* in cluster-c could be estimated using a subsidiary matrix and the circumstances of every student residing in every clustering center. The education leadership evaluation of a student, which is enhanced using environmental factors, is shown in equation (8). The student's progress is directly linked to influencing factors, and step-by-step improvements are expressed below:

(8) $$\begin{array}{c} P\left(C_{y}\right)=\frac{\prod_{y=0}^{N-1}\rho_{xy}\times Q_{st}\left(y\right)}{1+\prod_{y=0}^{N-1}\rho_{xy}}. \end{array}$$

*N* signifies the number of students, *Q*_*st*_ indicates the progress of the students' underneath the *y* factors involved, and *P*(*C*_*y*_) reflects the progress of the student *s*′ in cluster-c. The multiplication factor is indicated as *ρ*_*xy*_. Depending on which group the student belongs to, one may determine how well the student *st*′ performs under the variable *x*. The target leadership quality of a student is denoted in equation (9), and it shows the outcomes of the system. The final obtained prediction results of the education leadership of the student are shown below:

(9) $$\begin{array}{c} F\left({st}^{\prime },x\right)=\overset{N-1}{\underset{y=0}{\prod }}\rho_{xy}+\frac{1}{P\left(C_{y}\right)}. \end{array}$$

*ρ*_*xy*_ corresponds to a component of multiplier *ρ*, and *F*(*st*′, *x*) denotes the target learning performance underneath the factor *N*. *P*(*C*_*y*_) indicates the progress of students in the cluster *C*_*y*_.

The graphical representation of the function *F*(*st*′, *x*) is illustrated in Figure 3. The function uses the multiplier function *ρ*_*xy*_, and the progress of the education leadership of the students in the cluster *C*_*y*_ is denoted as *P*(*C*_*y*_). This function is used to analyze educational leadership improvement using FCM and big data algorithms.

### 3.4. Big Data Implications for Educational Leadership

The different environmental factors which affect the educational leadership quality of the students are analyzed by FCM and big data algorithm. The varying parameters to enhance the outcomes are shown below:

#### 3.4.1. Learning Benefits

For educational leaders, big data presents new learning opportunities. Educational leaders must familiarise themselves with these new resources and devices to successfully apply data-driven choices in the classroom context. They see how technology-based teaching methods account for most of the big data. In this situation, analytics can assist college principals in being more productive and effective in their research. Additionally, it enhances learning outcomes favorably. Students have more options for novel active learning due to using these tools. Students benefit from and broaden their knowledge by exchanging information with one another and with academic institutions. Educational institutions can use this information to address issues in education and prepare for the future.

The article "Influence Mechanism of Educational Leadership on Environmental Accounting Based on Big Data Algorithm" was retracted in 2023. Reasons: unreliable results or conclusions; concerns about the data; concerns about the peer review; concerns about the citations.

#### 3.4.2. Efficiency and Effectiveness in Decision Making

Making decisions is a complex process, whether individually or in groups. Leaders must make various decisions, including basic and complex ones, big and minor ones, programmable and nonprogrammer ones, technical and operational or practical judgments, and decisions involving individuals and groups. These decisions are made to pick the best options given the situation and raise the group's quality and efficiency. The “Big Data” notion can fundamentally alter how it conducts education by changing the modes of communication among learners and instructors and effectively meeting each learner's unique needs. Big data is a data system that college administrators utilize to make decisions about education. They can make decisions made by school administrators more efficient and successful.

The education leadership analysis system based on environmental accounting factors using big data is illustrated in Figure 4. The system uses FCM and environmental factors to detect and predict the students' education leadership. The big data modules help to provide the necessary data required for the survey and analysis. When using “Big Data” to make decisions, educational leaders gain several benefits. Here are a few big data benefits for school administrators in decision-making.

- *Effectiveness in Managing Tasks*. Without sound administrative decision-making, all of an academic institution's other responsibilities cannot be carried out as intended. Big data offers current information to decision-makers. This improves the effectiveness of leaders' managing duties
- *Beneficial for Development and Planning*. Making a decision is the initial step in constructing any plan. Big data offers an accurate study of history and can be applied to forecast the future. The planning and policy-making processes of any educational organization are improved when educational leaders have access to a wealth of information
- *Time Savings*. In today's cutthroat business environment, promptly selecting the best options is crucial to any corporation's success. Big data assists faculty members in various methods and enhances the performance and profitability of an academic institution's activities. Therefore, it is essential to the achievement of educational organizations

The article "Influence Mechanism of Educational Leadership on Environmental Accounting Based on Big Data Algorithm" was retracted in 2023. Reasons: unreliable results or conclusions; concerns about the data; concerns about the peer review; concerns about the citations.

### 3.5. Strategy Analysis Based on Big Data

The associated control approach is set following the correlation test for various indicators. Multiple elements of the analysis results are based on the cognitive control systems using different influencing environmental factors, as indicated in Table 1.

The different influencing factor that affects the education leadership of the student is analyzed, and the comparison results are shown in Table 1. The different influencing factors, namely, instructional design, platform function, social factor, and learning motion, help to increase the education leadership outcomes.

### 3.6. Policy Recommendations and Future Study

Understanding how educational leadership affects numerous receivers, including students, staff members, and teachers, is crucial. A clearer picture of what an instructional leader needs to do to strengthen their competencies, any weak points and collaborate on them for advancement, change management style, or embrace other management philosophies can be achieved by analyzing the impacts of teacher management via its essential parts, realizing the way and level of control that every activity in the feature of the educational leadership and its outcomes, and acknowledging which contribution is more essential.

Ultimately, leaders can behave more effectively, increasing the results of teacher management by acknowledging the impact of leadership elements in everyday operations and the effective interaction between them. Teachers and administrators find this valuable study in better comprehending the relevance of interactions between leader traits, behaviors, and styles and how they affect effectiveness. Via these contributions, leaders learn how to deal with the issues of the moment to enhance results, elevate and create better energy, be competitive, and adapt to the changes of the times.

While diverse leadership practices and styles yield different benefits for stakeholders in teacher management, personal characteristics are crucial. Therefore, the technique of successfully mixing them has better results. This is consistent with other research that concludes that influential leaders must be able to modify their approach depending on the scenario and environment to get the desired effects. Leaders must be conscious of their fields of expertise, including those who need to grow or partner with someone whose style complements their own.

All education providers, including students, educators, and admin, would be able to evaluate the comparative and correlative significance among each other of the leader's features, management styles, and behaviors regarding organizational outcomes. This is sensible and researches in the field on the composition and layout of a particular survey. The relative importance of every individual component's involvement in the results of leader behavior is explained by an assessment method that was appropriately applied to an original sample of all these receivers.

The article "Influence Mechanism of Educational Leadership on Environmental Accounting Based on Big Data Algorithm" was retracted in 2023. Reasons: unreliable results or conclusions; concerns about the data; concerns about the peer review; concerns about the citations.

The research focuses on finding the students' education leadership quality using a big data algorithm, fuzzy C-means model for cluster optimization, and environmental factors for improving the leadership quality. The different influencing factors, recommendations, and future implications are discussed in this section. The outcomes and findings of the system are enumerated in Section 4.

## 4. Outcome and Findings

Three hundred participants with 200 men and 100 women participants are considered for the analysis (https://data.world/datasets/school-leadership) [21]. The upgraded education method is used in the intervention class. In contrast, the standard online learning model has been used in the group: the different environmental factors and big data model with FCM help to improve the effectiveness of the ELM-BDA [22]. Students from other colleges in China conduct the survey, and the overall results are analyzed in this section.

The survey data characteristics are analyzed and shown in Table 2. The participants are selected from different colleges in China which include 200 boys and 100 girls. The students are chosen from the age of 20 to 30. The education qualification of the students varies from higher education and postgraduate. The ratio of the higher education and postgraduate is selected as 60 : 40. The leadership position of the students is chosen as lower, middle, higher, and superior with the ratio of 40 : 27 : 23 : 10. The education leadership using big data are analyzed for the different students, and the influencing factors which affect the administration are analyzed [23, 24].

The student leadership score analysis of the ELM-BDA system is depicted in Figure 5. Equation (10) is used to compute the student's educational leadership skill, and the different influencing factors are directly linked to the student's score.

(10) $$\begin{array}{c} F\left(S,t\right)=\overset{N-1}{\underset{i=0}{\prod }}\rho_{xy}+\frac{1}{P\left(C_{y}\right)}. \end{array}$$

The student selected is indicated as *S*, and the present time is shown as *t*. *ρ*_*xy*_ is expressed the available different environmental factors which affect educational leadership. The student's progress is indicated *P*(*C*_*y*_). And it is improved using different big data modules.

The article "Influence Mechanism of Educational Leadership on Environmental Accounting Based on Big Data Algorithm" was retracted in 2023. Reasons: unreliable results or conclusions; concerns about the data; concerns about the peer review; concerns about the citations.

There are four different students randomly selected from the available participants. The other environmental influencing factors such as class preview, classroom performance, attendance, out-of-class activities, operation, and final education leadership scores of the students are computed and shown. The student's education leadership is directly related to the environmental factors and the big data analytical module. The ELM-BDA system effectively analyses the system outcomes with score prediction and a mathematical model with a lesser computation error [25].

The influencing environmental factor analysis of the ELM-BDA system is shown in Figure 6. The different factors include teaching activities that help to directly impact the student leadership, an evaluation system that is used to analyze the student's leadership level and which can be further enhanced, a platform function to showcase their leadership quality, social aspect to express the education leadership outside the campus, and learning emotion factor to test the proposed ELM-BDA system. The data for the analysis is gathered from the site (https://data.world/datasets/school-leadership). It includes student achievement, student progress, student leadership level, discipline referral, attendance rate, satisfactory factor, influence factor, etc., for the analysis.

Equation (11) is used to find the influencing parameter matrix, and the environmental factors *β*_*xy*_ are directly linked to the student's predicted score.

(11) $$\begin{array}{c} F\left(S,i\right)=\overset{N-1}{\underset{i=0}{\prod }}\;\beta_{xy}\times \frac{P\left(C_{y}\right)}{N+1}. \end{array}$$

The different available environmental factors like classroom atmosphere, friends, teachers, available facilities in the school, management support to teachers and students, and teaching methods are considered for the analysis. The environmental factor is indicated as *β*_*xy*_. The progress factor is indicated as *P*(*C*_*y*_). And the total number of influencing factors that affect education leadership is shown as *N*. The proposed system with a big data algorithm helps to identify the education leadership quality present in the students and helps to motivate and improve them through different environmental factors and training [26, 27].

The mean and variance analyses of transformational leadership are analyzed using different transformational leadership factors such as idealized influencing factor, inspirational motivation factor, intellectual stimulation factor, and individualized consideration factor. Equation (12) is computed the leadership function *F*(*S*, *m*) where *m* is the transformational leadership skills, and the outcomes are linked to the progress function *P*(*C*_*y*_).

(12) $$\begin{array}{c} F\left(S,m\right)=\overset{N-1}{\underset{i=0}{\prod }}\;\frac{P\left(C_{y}\right)}{N+1}+\overset{N-1}{\underset{i=0}{\prod }}\propto_{i}. \end{array}$$

The progress function of a particular student is computed as *P*(*C*_*y*_). The total number of transformational leadership skills is denoted as *N*. The environmental factor which affects the transformation of leadership skills is expressed as ∝_*i*_. The results are plotted in Figures 7(a) and 7(b). The student performance of education leadership is computed according to the different transformational leadership, and the mean and standard deviation values of other factors are analyzed and plotted for minimum and maximum educational leadership quality among the students.

The article "Influence Mechanism of Educational Leadership on Environmental Accounting Based on Big Data Algorithm" was retracted in 2023. Reasons: unreliable results or conclusions; concerns about the data; concerns about the peer review; concerns about the citations.

The mean and variance analyses of the transactional leadership quality are analyzed, and the results are shown in Figures 8(a) and 8(b), respectively. The transactional leadership quality is analyzed according to idealized influence and inspirational motivation factors. Equation (13) analyzed the leadership function *F*(*S*, *d*) where *d* is the transactional leadership skills, and the transactional leadership factors are computed with optimum function *O*_*f*_.

(13) $$\begin{array}{c} F\left(S,d\right)=\frac{1}{\sum_{x=0}^{N-1}\left(\mu_{d}/N\right)+S_{d}}. \end{array}$$

The learning attribute for the decision-making skill of the student is indicated as *μ*_*d*_. The total skills considered for the decision-making is denoted as *N*, and the decision-making ability of the student is indicated as *S*_*d*_.

The students' educational leadership quality is enhanced using the students' leadership score prediction and big data analytical model. The minimum and maximum education leadership students are selected, and their performance is evaluated using different transactional leadership factors. Results are compared with each other with mean and standard deviation values.

The decision-making skill of the students is analyzed, and it is directly linked to education leadership. The students' decision-making skills are analyzed based on the idealized influence factor and inspiration leadership skills motivation factors, and the comparison results are shown in Figures 9(a) and 9(b), respectively. The education leadership skills of the student *F*(*st*′, *x*) are analyzed using equation (9), where *x* is the decision-making skills, and the outcomes of the progress are indicated using the function *P*(*C*_*y*_). Using equation (8), the students' education leadership quality can be increased mainly by decision-making skills. The ELM-BDA system with the big data algorithm and leadership score prediction model using different influencing environmental factors ensure the ELM-BDA system's effectiveness in improving the participants' le.

The article "Influence Mechanism of Educational Leadership on Environmental Accounting Based on Big Data Algorithm" was retracted in 2023. Reasons: unreliable results or conclusions; concerns about the data; concerns about the peer review; concerns about the citations.

The ELM-BDA system is analyzed in this section to showcase the education leadership and the impacts of the different environmental influencing factors and big data algorithms. The leadership score prediction model with mathematical expression helps to reduce the error and help the student to develop their educational leadership skills at any point.

Figure 10 shows the student's knowledge level of environmental accounting. The research model recommends that the environmental accounting and educational leadership were given to learners with primary accounting education have an influence on the level of knowledge about the environmental laws, environmental data, and environmental accounting of the students and thus constitutes an ecological realization in the learners. There is an association between students who received environmental accounting education and knowledge about ecological data, environmental accounting, and environmental law. Correlation is a statistical technique utilized to identify the degree and direction of the connection between variables, regardless of whether the variables are dependent or independent.

The ELM-BDA system is analyzed in this section to showcase the education leadership and the impacts of the different environmental influencing factors and big data algorithms. The leadership score prediction model with mathematical expression helps to reduce the error and help the student to develop their educational leadership skills at any point.

## 5. Conclusion and Findings

This study presents the educational leadership model based on big data algorithm (ELM-BDA) to explore student leadership performance considering the environmental accounting notion. Big data tools assist school administrators' decision-making in the proper and timely manner. Big data might shape a cutting-edge, dynamic sch. The decision-making challenges that educational leaders experienced in the past will not exist in the new phase of “Big Data.” They would be capable of making it faster and more precisely. However, to fully benefit from big data, school administrators must adapt to mastering new big data techniques.

Colleges must deal with the vast amount of educational material that must be processed to maintain development, and they urgently need to improve the intelligence of their educational management. The study suggests an educational leadership model based on big data algorithm (ELM-BDA) to analyze the student leadership performance that relies on cooperative filtration and fuzzy C-means (FCM) and big data. This research evaluates the environmental factors and their impact on students' leadership skills.

The article "Influence Mechanism of Educational Leadership on Environmental Accounting Based on Big Data Algorithm" was retracted in 2023. Reasons: unreliable results or conclusions; concerns about the data; concerns about the peer review; concerns about the citations.

Additionally, level curriculum ranging this big data to make smart decisions enables school administrators to enhance classroom instruction. By merging various information and telecommunication platforms, big data facilitates efficient decision-making for the school system and improves students' leadership skills. The future need for developing more learning control systems by academic institutions increases due to this trend to efficiently use big data for decision-making.

Moreover, there is an opportunity for improving the offered algorithm's operational efficiency. The issues mentioned above will be resolved through further research. This study is aimed at providing crucial technical assistance so that higher education administration can be more innovative, waste less labor, and enhance the student's leadership skills.

## Figures and Tables

**Figure 1:** The FCM clustering model for educational leadership on environmental accounting.

**Figure 2:** The student education leadership performance analysis based on environmental accounting factors.

**Figure 3:** The graphical representation of *F*(*st*′, *x*).

**Figure 4:** The education leadership analysis system based on environmental accounting using big data.

**Figure 5:** Student leadership score analysis

**Figure 6:** Influencing environmental factor analysis of the ELM-BDA system

**Figure 7:** (a) Mean analysis of transformational leadership. (b) Variance analysis of transformational leadership.

**Figure 8:** (a) Mean analysis of transactional leadership. (b) Variance analysis of transactional leadership.

**Figure 9:** (a) Mean analysis of decision-making leadership. (b) Variance analysis of decision-making leadership.

**Figure 10:** Student knowledge level about environmental accounting

**Table 1:** Influencing factor analysis.

Component inducing movement	Initiative	Control strategy
Instructional layout	Actions to instruct and ways to teach	Need to be wealthy, and move learning resources introduced by various organizations or media based on how you learn best.
	Review process scheme	Must be enhanced

The task of a framework	Assistive technology for education	The learner's present development level can be depicted visually. Observe how students in your class are progressing in their studies. Learners' development compared to usual progress can be shown as a gap. Inform the slow people.

Cultural viewpoint	Trainer and students	Encouraging and reminding students who receive little or no attention

Emotional literacy	Learning data	Students' academic achievements can be visualized. Analyze the existing class's or status' overall score if possible. Think about how the learners in the existing group or rating compare to each other.

The article "Influence Mechanism of Educational Leadership on Environmental Accounting Based on Big Data Algorithm" was retracted in 2023. Reasons: unreliable results or conclusions; concerns about the data; concerns about the peer review; concerns about the citations.

**Table 2:** Survey data characteristics.

Characteristics	Variants	Count	Percentage
Gender	Male	200	67
	Female	100	33

Age	Below 20	50	17
	20-25	86	29
	25-30	82	27
	Above 30	82	27

Education	Higher	180	60
	Postgraduate	120	40

Leadership position	Lower	120	40
	Middle	80	27
	Higher	70	23
	Superior	30	10

## Data Availability

The data that support the findings of this study are available from the corresponding author upon reasonable request.
